The article "Pop Music Trend and Image Analysis Based on Big Data Technology" was retracted in 2023. Reasons: signs of a paper mill; suspected computer-generated content; unreliable results or conclusions; concerns about the data.

# Pop Music Trend and Image Analysis Based on Big Data Technology

**DOI:** 10.1155/2021/4700630

**Published:** 2021-12-09

**Authors:** Jinyan Ren

**Affiliations:** Conservatory of Music Shanxi University, Taiyuan, Shanxi 030006, China

## Abstract

With people's pursuit of music art, a large number of singers began to analyze the trend of music in the future and create music works. Firstly, this study introduces the theory of music pop trend analysis, big data mining technology, and related algorithms. Then, the autoregressive integrated moving (ARIM), random forest, and long-term and short-term memory (LSTM) algorithms are used to establish the image analysis and prediction model, analyze the music data, and predict the music trend. The test results of the three models show that when the singer's songs are analyzed from three aspects: collection, download, and playback times, the LSTM model can predict well the playback times. However, the LSTM model also has some defects. For example, the model cannot accurately predict some songs with large data fluctuations. At the same time, there is no big data gap between the playback times predicted by the ARIM model image analysis and the actual playback times, showing the allowable error fluctuation range. A comprehensive analysis shows that compared with the ARIM algorithm and random forest algorithm, the LSTM algorithm can predict the music trend more accurately. The research results will help many singers create songs according to the current and future music trends and will also make traditional music creation more information-based and modern.

## 1. Introduction

As an entertainment product, pop music has attracted more attention. According to relevant research, China's mobile music market developed rapidly from 2013 to 2018. In addition, the development of many types of popular music determines the main development direction of music in the future to a certain extent [1]. It reflects the influence of many social behaviors on pop music and the audience's preference for related music [2, 3]. Using image analysis and prediction of the development trend of pop music, the collection of resources in the music library, and the integration of user behavior on different platforms, we can analyze user data and preferences, provide various pop music data sets, accurately analyze the specific attributes of music works, and accurately control dynamic pop music. The trend of user preferences determines the form of pop music [4]. There is little research on the image prediction of pop music trend all over the world. Alibaba Group launched Alibaba music trend forecast in 2016. After approximately 7 years of development, Alibaba music has nearly 1 million analysis records and historical user behavior data. Later, the number of artists or songs to be played in the next step and the future dark horse will be excluded from the mainstream data. Multiple music platforms will mainly control the trend of pop music [5].

Data mining is a new discipline born in the 1980s. It is mainly oriented to the research field of artificial intelligence for business applications. From a technical point of view, data mining is a process of obtaining implicit, undetected, and potentially valuable information and knowledge from a large number of complex, irregular, random, and fuzzy data. Data mining is to extract, transform, and analyze some potential laws and values from a huge database to obtain key information and useful knowledge to assist business decision-making. Today, more than 90% of the data on the internet is generated within two years, and the amount of data generated every day is still rising with great ease. Under this background, it is not enough to have the ability to receive and store massive data alone. It is also necessary to deal with these data effectively to obtain the laws and patterns that can guide the future behavior and improve the efficiency of enterprises, society effectiveness, and efficiency of organizations and institutions. The speed of computer processing is very fast, however, the law of digging and saving from massive data broadcasting is not a simple operation. Therefore, it is necessary to have a good data mining algorithm to complete the process of “gold in the sand.” Therefore, various data digging and saving algorithms came into being.

The current research aims to predict the music trends using the LSTM (long-term and short-term memory) algorithm and big data technology images, and they help the singers create songs according to the current and future trends of pop music. The innovation of this study is to select the most appropriate and accurate algorithm model by the comparative analysis of the ARIM algorithm, random forest algorithm, and LSTM algorithm. The results show that compared with the traditional image prediction model, the LSTM algorithm has a better prediction accuracy.

## 2. Related Works

In the current era of big data, various industries try to get rid of traditional development modes by utilizing data. The music industry has gradually aroused numerous scholars' interest in studying the application of big data in this field.

Wang et al. proposed a CL-LDA (Latent Dirichlet Allocation) topic model that could well adapt to the topic mining task of short text with sparse semantics and a lack of cooccurrence information in OHCs (online health communities) [6]. Hervé et al. found that the extraction of semantic memory and situational memory was completed by different neural networks. However, these results were basically obtained using language and visual space materials. They tried to utilize common or uncommon melodies to explore the neural substrates under the semantic and episodic elements of music [7]. Jin et al. designed a smart neural network for music composition to automatically create specific genres of music. The model had a superior and innovative structure that acquired the music sequence using an actor's long short-term memory. Then, it decided the probability of the sequence by a procedure via reward as feedback to improve the performance of music creation. Besides, the rule of music theory was introduced to confine the genre of generated music [8]. Pelchat and Gelowitz input the images of spectrograms generated from the time slices of songs into a neural network to classify the songs into their respective musical styles [9]. Yan trained the network weights by the T-S-based cognitive neural network and improved the genetic algorithm. They integrated the integration of the momentum method and learning rate-adaptive adjustment with the membership function parameter adjustment strategy. Besides, they introduced a compensation factor correlated to the input dimension into the membership degree. The extreme input dimension resulted in rule calamity, indicating that their research method was suitable for the music recognition system [10]. Meng and Chen selected two methods different from the previous Mel Cepstral Coefficients and Constant *Q* Transform to extract the features of music, and they used the convolution neural networks for training and recognition. They adopted the Mel cepstral coefficient to determine timbre and used the constant *Q* transform to determine pitch. They finally found that the recognition success rate reached 95% after inputting the corresponding features into the neural network for training and learning [11]. Zhang et al. proposed an improved music separation method based on discriminative training depth neural network and presented an improved objective function to discriminate against the training. Moreover, they added an additional layer to the DNN model and introduced the time-frequency masking to optimize the estimated accompaniment of the song. They obtained the corresponding time-domain signal using inverse Fourier transform. Finally, they verified the influence of different parameters on the separation performance and compared it with the existing music separation methods. Their experimental results showed that the improved objective function and the introduction of time-frequency masking significantly improved the separation performance of the DNN, and the separation performance improved by approximately 4 dB compared with other existing music separation methods [12]. Dawson et al. stated that people could train the networks to solve musical problems and study how these networks encode musical properties. They also reported very high correlations between the network connection weights and discrete Fourier phase spaces used to represent the musical sets [13]. Dorfler et al. posed the question of whether replacing it by applying adaptive or learned filters directly to the raw data can improve learning success. The theoretical results showed that approximately reproducing the mel-spectrogram coefficients by applying the adaptive filters and subsequent time-averaging on the squared amplitudes was in principle possible. They also conducted extensive experimental work on the task of singing voice detection in music. The results of their experiments showed that for the classification based on convolutional neural networks, the features obtained from the adaptive filter banks followed by time-averaging the squared modulus of the filters' output perform better than the canonical Fourier transform-based mel-spectrogram coefficients. They believed that the alternative adaptive approaches with center frequencies or time-averaging lengths learned from the training data performed equally well [14]. Liu et al. exploited the low-level information from the spectrograms of audio and developed a novel CNN architecture that took the multiscale time-frequency information into consideration. The CNN architecture transferred more suitable semantic features for the decision-making layer to discriminate the genre of the unknown music clip. They conducted experiments on the benchmark datasets, including GTZAN, Ballroom, and Extended Ballroom, which proved the excellent performance of the architecture [15]. Zhou established the database of regional culture and music characteristic resources by data mining technology and classified the regional characteristic music and cultural resources data combined with the improved BP (Back Propagation) neural network model. They also constructed a set of databases including classification, search, audition, and storage to protect and spread the regional music characteristic cultural resources. At the same time, it also provides new ideas for cultural heritage [16].

The above research on big data and different neural networks in the field of music has promoted the maturity of these technologies. There are certain differences in the accuracy of music prediction models established by different types of neural networks and algorithms applied in the field of music. Therefore, different algorithms are selected to establish models here to predict the music trend more accurately.

## 3. Construction of Prediction Models and Scheme Design

### 3.1. Analysis of the Music Trend

A group of people in society, driven by certain psychological needs, carry out certain music behavior in a certain period, resulting in a certain music genre spread in a certain social background. This social phenomenon may form different degrees of social popularization and social fanaticism, which can be called music popularization. The music trend here is limited to a singer's specific distribution point in future.

The current analysis and research of music are mainly under the foundation of users' advice. There are few studies in the field of pop music teaching, including neural networks, Gaussian mixture model, and support vector machine. The commonly used prediction methods of music ending prediction contain the SVM (support vector machine) and ANN (artificial neural network). These models generally have a limited learning ability and a high-dimensional kernel function with low explanatory ability. In particular, the radial basis function is sensitive to missing data [17], which is not a good choice for processing the mass of online music data. The utilization of artificial neural networks to build a music trend prediction model requires a large experimental environment and a long time with a medium prediction effect. Additionally, the artificial neural network needs various parameters that have great influences on the experimental results and bring complex workload [18]. The network music data is diverse, complex, high dimensional, and considerable. The existing music video model and the traditional statistical model are often difficult to realize the efficient data analysis of online songs (downloads, play count, and collections). Moreover, musicians have many difficulties in connecting with audiences. The results of the deep mining of music data are not ideal either. In recent years, many prediction models have been studied from the perspective of regression prediction and time series. They have achieved prediction results with a relatively high accuracy based on the Random Forest algorithm in many areas. Therefore, according to the regression prediction method, the ARIM algorithm, Random Forest algorithm, and LSTM algorithm are selected to establish the prediction models of music trend from the perspective of time series prediction.

### 3.2. Big Data Mining

Figure 1 shows the CRISP-DM (cross-industry standard process for data mining) reference model. In the process of data mining, there are two vital links, namely, model evaluation and model establishment, both of which belong to machine learning.

Machine learning is a process of computers' simulation of human learning behavior. As two foundations of data mining, machine learning provides technical methods for analyzing data, and the database technology realizes the data management of data mining.  Figure 2 represents the nexus of database technology, data mining, and machine learning [19]. There are three main types of machine learning: semisupervised learning, unsupervised learning, and supervised learning.

Supervised learning involves a set of labeled data, enabling computers to use specific patterns to identify the new samples of each labeled type. The two main types of supervised learning are classification and regression. The representative methods of supervised learning include the decision tree, Naive Bayes model, and support vector machine. In unsupervised learning, the data is labelless like most data in the real world. Hence, the unsupervised learning algorithm is particularly useful [20]. Unsupervised learning methods are divided into two categories: (1) one is a direct method based on the probability density function estimation: trying to find the distribution parameters in the feature space and classifying them. (2) The other is the concise clustering method based on the similarity measure between the samples: its principle is to try to determine the core or initial core of different categories and aggregate the samples into different categories according to the similarity measure between the samples and cores. Using the clustering results, we can extract the hidden information in the data set, classify the future data, and predict the future data. It is applied to data mining, pattern recognition, image processing, etc. The clustering is mainly used to classify the data according to its behavior or attribute, while the dimensionality reduction can reduce the variables of data sets. The most representative of unsupervised learning is the K-Means method. The role of semisupervised learning is to classify the data with or without labels using the classification function. The most representative algorithm of semisupervised learning is the expectation maximization algorithm [21].

### 3.3. Regression Analysis Model

#### 3.3.1. Random Forest Algorithm

Random forest refers to a classifier that uses multiple trees to train and predict samples. Random forest is an algorithm that integrates multiple trees using the idea of ensemble learning. Its basic unit is the decision tree, and its essence belongs to a major branch of machine learning—ensemble learning method. There are two keywords in the name of random forest, one is “random” and the other is “forest.” Machine learning can usually be divided into the following categories: dimension reduction, clustering, regression, and classification. Regression is not only a kind of supervised learning technology but also a relatively comprehensive technology. The main role of regression is to predict targets, such as future weather, future stock markets, or commodity prices. Compared with other methods, regression is the highest prediction method in terms of accuracy. Therefore, many studies use the regression model to predict and analyze related issues. The most appropriate method should be selected first in the process of establishing the regression model. For example, the least square method is suitable when the dimension of the surveyed data is relatively small [22]. The regression model is widely applied in a vast range of prediction fields, such as the stock trend, economic trend, future product sales, and event risk prediction. Besides, the collaborative Random Forest algorithm can also have good prediction effects and broad applicability. The Random Forest algorithm is essentially a type of supervised learning algorithm, which is an integrated learning algorithm by a decision tree. The Random Forest algorithm can be applied not only to the classification of problems but also to the regression model [23].

#### 3.3.2. Decision Tree Algorithm

The decision tree is a tree structure in which each internal node represents a test on an attribute, each branch represents a test output, and each leaf node represents a category. The classification tree (decision tree) is a very common classification method. It is a kind of supervised learning. The so-called supervised learning is that given a pile of samples, each sample has a set of attributes and a category. These categories are determined in advance, and then, a classifier can be obtained by learning, which can give correct classification to the new objects.  Figure 3 shows the decision tree, where the circle represents the root node and internal node, and the square represents the leaf node.

Three steps must be followed in the process of establishing a decision tree. Firstly, select the features of the target object. Secondly, establish the growth trend of the tree. Thirdly, prune the tree. So far, the decision tree algorithm has been widely used in stock prediction, commodity price prediction, housing price forecast, and the prediction of future economic trend. It has achieved excellent achievements in many fields.

(1) Entropy: the essence of entropy is to interpret the uncertainty in random variables. Let *X* be a random variable and the value of *X* be a range of *X*_1_, *X*_2_,…, *X*_*n*_. *X*_*i*_ represents the values that may be taken, and the probability that the random variable *X* equals *X*_*i*_ is set as *P*_*i*_. Then, set the entropy of random variable *X* as *H*(*X*), which can be written as

(1) $$\begin{array}{c} H\left(X\right)=-\sum_{i=1}^{n}p_{i}\log_{2}p_{i}. \end{array}$$

Let *D* be the sample set. The random variable *X* represents the specific category of *D*. There are a total of *K* categories in the selected sample *D*. Meanwhile, |*C*_*K*_| denotes the number of samples of category *K*, and |*D*| is the total number of samples. Then, the probability of each category is *CKD*, and the entropy of the sample set *D* is expressed as

(2) $$\begin{array}{c} H\left(D\right)=-\sum_{K=1}^{K}\frac{\left|C_{K}\right|}{\left|D\right|}\log_{2}\frac{\left|C_{K}\right|}{\left|D\right|}. \end{array}$$

(2) Information gain: the information gain is the difference value of entropy before and after the data set is divided by a feature. The essence of entropy represents the uncertainty in the random variables. When the value of entropy increases, the uncertainty of variables in the sample will also increase. Therefore, the difference value of entropy before and after the division can be used to judge the division effect of the sample set *D* in the current feature. The entropy of the sample set *D* before the division is certain. The information gain *g* (*D*, *A*) is equal to the difference between the entropy *H*(*D*) before the division of data set *D* by a feature *A* and the entropy *H*(*D*) of *D*. The calculation of *g* (*D*, *A*) is shown as

(3) $$\begin{array}{c} g\left(D,A\right)=H\left(D\right)-H_{A}\left(D\right). \end{array}$$

(3) Information gain ratio: the information gain ratio is the product of a penalty parameter *P* and the information gain in essence. The penalty parameter is the reciprocal of the entropy *H*_*A*_(*D*) of the data set *D* with feature *A* as a random variable; that is, the samples with the same value of feature *A* are divided into the same subset. In general, the penalty parameter is inversely proportional to the number of features.

The penalty parameter can be calculated as follows:

(4) $$\begin{array}{c} P=\frac{1}{H_{A}\left(D\right)}. \end{array}$$

Equation (5) is the calculation method of information gain ratio:

(5) $$\begin{array}{c} g_{R}\left(D,A\right)=\frac{g\left(D,A\right)}{H_{A}\left(D\right)}, \end{array}$$

In the above equation, *H*_*A*_(*D*) is the entropy obtained by taking the current feature *A* as the random variable for the sample set *D* and *g* (*D*, *A*) represents information gain.

#### 3.3.3. Linear Regression Algorithm

Suppose there is a data set and substitute some features *X*_1_, *X*_2_,…, *X*_*P*_ to predict the object variable *Y*. In a relatively simple model, it is assumed that the object variable *Y* is a linear combination of these features:

(6) $$\begin{array}{c} y\approx a_{0}+a_{1}x_{1}+\cdots +a_{p}x_{p}. \end{array}$$

### 3.4. Time Sequence Model

#### 3.4.1. LSTM Model

LSTM is a special RNN (Recurrent Neural Network) structure that is improved based on RNN [24]. LSTM itself is a part of the whole neural network rather than an independent network structure, replacing the hidden layer units in the original network. LSTM can deal with the data with “sequence” properties like time series data, such as daily stock price trend and time domain waveform of mechanical vibration signals. Also, it can process data like the data of natural language with sequence properties consisting of ordered words [25].

All RNNs have a chain with repetitive neural network modules. In the standard RNN, this repetitive structural module has only one very simple structure, such as a tanh layer. LSTM is also such a structure, but the repetitive modules have different structures. Different from the structure of a single neural network layer, there are four interaction layers in LSTM, which interact in a very special way. LSTM is an artificial RNN architecture for deep learning [26].

LSTM can not only process a single data point (such as image) but also process the whole data sequence. The LSTM unit consists of memory unit, input gate, output gate, and forget gate. The memory unit can remember the values within any time interval, and the three gates control the information flow entering or existing the unit. LSTM is especially suitable for the classification, processing, and prediction of time series data because there may be a lag of unknown duration between the important events in a time series. LSTM is developed to deal with the explosion and disappearance gradient problems that may occur in the training of traditional RNNs. The relative insensitivity to gap length is the advantage of LSTM over the RNN, hidden Markov model, and other sequential learning methods in many applications.

The first step in LSTM is to decide what information to discard from the cell state, which is completed using the forget gate. The role of the input gate is to add new data to the cell state. The role of the output gate is to determine the value of the output. *X*_*t*_ represents the input, *S*_*t*−1_ denotes the unit of state memory, and *h*_*t*−1_ signifies the intermediate output in the forget door. The retained vector in the updated state memory unit is determined jointly by *X*_*t*_ under the action of sigmoid function and tanh function. Moreover, *s*_*t*_ represents the state of the memory unit after being updated, while *o*_*t*_ stands for the state of the output gate, and *h*_*t*_ refers to the intermediate output. Then, equations (7)–(12) are obtained:

(7) $$\begin{array}{c} f_{t}=\sigma \left(W_{fx}x_{t}+W_{fh}h_{t-1}+b_{f}\right), \end{array}$$

(8) $$\begin{array}{c} i_{t}=\sigma \left(W_{ix}x_{t}+W_{ih}h_{t-1}+b_{i}\right), \end{array}$$

(9) $$\begin{array}{c} g_{t}=\phi \left(W_{gx}x_{t}+W_{gh}h_{t-1}+b_{g}\right), \end{array}$$

(10) $$\begin{array}{c} O_{t}=\sigma \left(W_{ox}x_{t}+W_{oh}h_{t-1}+b_{o}\right), \end{array}$$

(11) $$\begin{array}{c} s_{t}=g_{t}⊙i_{t}+s_{t-1}⊙f_{t}, \end{array}$$

(12) $$\begin{array}{c} h_{t}=\phi \left(s_{t}\right)⊙O_{t}. \end{array}$$

Among the above equations, *f*_*t*_ is the state of the forget gate, while *i*_*t*_ represents the state of input gate, and *g*_*t*_ denotes the input node. Besides, *o*_*t*_ refers to the state of output gate, *s*_*t*_ is the state memory unit, and *h*_*t*_ represents the state of intermediate output. *W*_*fx*_, *W*_*ix*_, *W*_*gx*_,  and *W*_*ox*_ are the matrix weights of the forget gate, input gate, input node, and output gate multiplied by input *x*_*t*_, respectively. Meanwhile, *W*_*fh*_ denotes the forget gate, while *W*_*ih*_ represents the input gate, and *W*_*gh*_ is the input node. Besides, *W*_*oh*_ represents the weight of the matrix after the multiplication of the intermediate output *h*_*t*−1_ and the output gate. Furthermore, *b*_*f*_, *b*_*i*_, *b*_*g*_, and *b*_*o*_ are the bias items of the forget gate, input gate, input node, and output gate, respectively. Meanwhile, ⊙ represents the multiplication of each element in the vector by bit, *σ* denotes the change of sigmoid function, and Φ represents the change of tanh function.

#### 3.4.2. ARIMA (Autoregressive Integrated Moving Average) Model and ARMA (Auto-Regressive and Moving Average) Model

In the process of time series research, the ARIMA model is the optimization of ARMA model [27–29]. Both models are suitable for processing time series data. The ARIMA model can achieve the accurate prediction of data. When the obtained data features are not very stable, the ARIMA model can be used to steady the data features using the initial difference method [30–32].

### 3.5. Analysis of Data Feature

1. Distribution analysis: firstly, under the premise of ensuring the data quality, tools, such as drawing software, programming software, modeling software, and analysis software, are used to visualize the song data to further observe the distribution of the data. The specific types and characteristics of the data can be obtained by the analysis of data distribution. If the obtained data are quantitative data, then the distribution histogram and frequency distribution table are established to visually present the data. Otherwise, the bar chart, pie chart, and line chart are drawn to realize the visualization of qualitative data.
2. Comparative analysis: the comparative analysis of the obtained relevant indicators in the perspective of data amount can evaluate the prediction accuracy of the algorithm. The comparative analysis can also be conducted on data distribution, which is usually used for the comparison analysis of time series and the horizontal or vertical comparison between different indicators. For example, using horizontal and vertical comparative analysis from the three aspects of the play count, collection, and downloads of a song, singers can be divided into two types: exploding singers and stable singers.
3. Statistical analysis: this method mainly analyzes data distribution, such as distribution shape analysis, dispersion degree detection, and concentration analysis. The basic statistics describing data are also divided into three categories: distribution shape statistics, dispersion statistics, and central tendency statistics. The statistics and analysis of the data of every song is presented in the form of graphs to further study the distribution rules and data trends. The following three statistics are used to identify and analyze the data: collection, downloads, and play count.

## 4. Data Processing and Predictive Analysis

### 4.1. Prediction Results of LSTM Model

Figure 4 illustrates the statistics of collection, play count, and downloads of different types of singers.

The LSTM model is used to compare the real and predictive values of three singers from mainland China, Hong Kong, and another country, as shown in Figure 5.

Upon the comparison of the real value and predictive value of three singers from different places, the prediction error of the singer from mainland China is relatively large. However, the prediction of the other two singers is basically close to the actual value. Meanwhile, the prediction data fluctuates violently overall, but it will eventually stabilize and come close to the real value.  Figure 6 presents the statistics of collection, downloads, and play count of nine songs, including three Chinese songs, three Cantonese songs, and three English songs.  Figure 7 shows the prediction value and actual value of the play count of the nine songs.

Upon the prediction of nine songs from the collection, downloads, and play count, the model achieves a good prediction of the play count of the nine songs on the whole. However, the model cannot accurately predict the play count of the songs with wide fluctuations. The prediction results of other aspects are basically close to the actual situation. Therefore, the prediction of music trend by the time series of LSTM algorithm shows a good effect.

### 4.2. Prediction Results of the ARIMA Model

Figure 8 represents the comparison of the play count of two songs of different singers.

According to Figure 8, the daily playing count of the songs of the two singers is close to the stationary time series. Therefore, the first-order difference operation is performed on the data of the play count to make the original time series data with large fluctuations become relatively stable time series data.  Figure 9 illustrates the prediction of the play count of a song in the next two months from the perspectives of users and singers.

Figure 9 shows that there is no obvious gap between the predictive value of the play count of the song and the actual value, and the error fluctuation of predictive value is within the allowable range. Therefore, the ARIMA model can accurately predict the play count of songs.

### 4.3. Comparison of Prediction Results of Different Models

In the experiment, the model predictions of the rim algorithm, random forest algorithm, and LSTM algorithm are compared.  Figure 10 illustrates the MAE (mean absolute error) and RMSE (root mean square error) of the prediction results. From October 1, 2020, to October 31, 2020, the test predicts the playback times of the nine songs using the ARIM algorithm, random forest algorithm, and LSTM algorithm.

According to Figure 10, the LSTM algorithm has a better prediction performance in the play count of songs of the nine artists than the ARIM algorithm and Random Forest algorithm. Besides, compared with the other two algorithms, the RMSE and MAE of the LSTM algorithm have reduced the data from 0.072 and 0.045 to 0.045 and 0.032, respectively. Meanwhile, the error rate is reduced by 36.5% and 28.1%, compared with the ARIM algorithm and the Random Forest algorithm. Therefore, the LSTM algorithm can predict the music trend more accurately.

## 5. Conclusion

The prediction of music trend is mainly achieved by the LSTM and big data mining. The prediction models are established by the ARIM algorithm, Random Forest algorithm, and LSTM algorithm to predict the data of songs and calculate the fluctuation of time series. The results show that after analyzing the nine singers' collection, downloads, and play count, the LSTM model makes a good prediction on the play count of the nine singers' songs. However, there are also some defects in the LSTM model. For example, the model cannot accurately predict for some songs with large data fluctuations. The prediction results of other aspects are close to the actual situation.

Meanwhile, there is no big error in the play count of prediction results of the ARIM algorithm and the actual value, and the error fluctuation of the prediction is also within the allowable range. This indicates that the ARIM algorithm can also meet the prediction analysis. After comprehensive analysis, the LSTM algorithm has the most accurate prediction of the music trend among three algorithms. However, there are still some defects in this study. As songs usually have a relatively high periodicity and randomness and are greatly affected by the external factors, it is possible that the emergence of some film and television works can lead to a dramatic increase in the play count of music. Therefore, the feasibility error analysis of these aspects should be carried out in future research.

## Figures and Tables

**Figure 1:** CRISP-DM reference model.

**Figure 2:** Nexus of database technology, data mining, and machine learning.

**Figure 3:** Decision tree.

**Figure 4:** Statistics of play count, downloads, and collection of singers: (a) stable singers and (b) exploding singers. (A) Play count, (B) downloads, and (C) collection.

**Figure 5:** Comparison of the actual value and predictive value of LSTM model: (a) singer from Mainland China, (b) a Hong Kong singer, and (c) a foreign singer.

**Figure 6:** Statistics of play count, downloads, and collection of nine songs: (a–c) a singer from mainland China, (d–f) a Hong Kong singer, and (g–i) a foreign singer.

**Figure 7:** Comparison of the predictive value and actual value of play count of nine songs: (A) predictive value and (B) actual value. (a–c) A singer from mainland China, (d–f) a Hong Kong singer, and (g–i) a foreign singer).

**Figure 8:** The play count of two songs (A and B are two different singers).

**Figure 9:** Comparison of predictive value and actual value of the play count (A: actual value; B: predictive value).

**Figure 10:** Prediction results of different models: (a) RMSE and (b) MAE. (A) LSTM algorithm, (B) ARIM algorithm, and (C) random forest algorithm.

## Data Availability

The data used to support the findings of this study are available upon request to the author.
